# Encapsulation of Liposomes within pH Responsive Microspheres for Oral Colonic Drug Delivery

**DOI:** 10.1155/2012/458712

**Published:** 2012-06-27

**Authors:** M. J. Barea, M. J. Jenkins, Y. S. Lee, P. Johnson, R. H. Bridson

**Affiliations:** ^1^Centre for Formulation Engineering, School of Chemical Engineering, University of Birmingham, Edgbaston B15 2TT, UK; ^2^School of Metallurgy and Materials, University of Birmingham, Edgbaston B15 2TT, UK; ^3^School of Cancer Sciences, University of Birmingham, Edgbaston B15 2TT, UK

## Abstract

A novel liposome-in-microsphere (LIM) formulation has been created comprising drug-loaded liposomes within pH responsive Eudragit S100 microspheres. The liposomes contained the model drug 5-ASA and were coated with chitosan in order to protect them during encapsulation within the microspheres and to improve site-specific release characteristics. *In vitro* drug release studies showed that LIMs prevented drug release within simulated stomach and small intestine conditions with subsequent drug release occurring in large intestine conditions. The formulation therefore has potential for oral colonic drug delivery.

## 1. Introduction

Within oral drug delivery, specific targeting of the colon can be advantageous due to near-neutral pH, low enzyme and bile salt activity and long residence time. For local treatment of colonic diseases, direct targeting may increase drug bioavailability at the target site, therefore allowing reductions in administered dose and systemic side effects [1]. It has also been shown that specific targeting to the colon is advantageous for systemic treatments for a number of reasons including the potential for protein and peptide drug absorption [1, 2]. However, oral drug delivery to the colon is associated with a number of obstacles including dosage form transit through regions of high acidity and digestive activity. 

Liposomes are drug carriers that can be used for a wide range of active ingredients [3], have the ability to interact with cells [4], and have potential in gene transfection [5]. Evidence also suggests that they can advantageously interact with colonic tissue and/or find utility in colonic drug delivery [6–9]. However there is little information on how they could be delivered to this region, particularly via the oral route, which is generally the favoured route for drug administration. Liposomes are not naturally suited to oral drug delivery due to their susceptibility to digestion en route through the GI tract. Coating them with a polymer is one way that may protect them during transit, but very little work has been done on specifically targeting the colonic region. 

Previously, we have described the direct coating of liposomes with the methacrylic acid copolymer Eudragit S100, as a means to facilitate colonic targeting following oral administration [10]. With its anionic carboxylic acid side groups and solubility threshold of pH 7, the Eudragit S100 coat allowed an appropriate pH-dependent drug release profile to be achieved, but the coat was not able to prevent ingress of bile salts, which would lead to premature drug release *in vivo*. The aim of the current work was therefore to improve that formulation and to create a novel liposome-in-microsphere (LIM) system comprising chitosan-coated liposomes surrounded by a solid shell of Eudragit S100. Chitosan, as a polymer resistant to the organic solvents used in microsphere production, was included to protect the liposomes during their encapsulation. Chitosan is also known to be solubilised by the specific polysaccharidases (glucosidases, glycosidases), which are secreted by colonic bacteria, through the random scission of the 1,4 glycosidic bond [11, 12]. Therefore its incorporation would also facilitate colonic targeting via a mechanism discrete to that imparted by the Eudragit S100. Given that inter- and intrapatient variation in gastrointestinal (GI) tract conditions (particularly pH) can be significant, formulations reliant on more than one physiological trigger may provide a more accurate means of delivery to the colon [13]. 

## 2. Materials and Methods

### 2.1. Materials

Liposomal membrane components included egg phosphatidylcholine (EPC) (a gift from Lipoid, Ludwigshafen, Germany, minimum 98% purity), cholesterol (CH) (Sigma Aldrich, Dorset, UK), and dicetyl phosphate (DCP) (Sigma Aldrich). 5-aminosalicylic acid (5-ASA)(Sigma Aldrich) was chosen as it is an anti-inflammatory drug used in the treatment of ulcerative colitis and Crohn's disease. Chitosan (low molecular weight measured at 237,000 by gel permeation chromatography, Sigma Aldrich) was used to coat the liposomes. Eudragit S100, the pH responsive polymer used for producing the microspheres, was a gift from Evonik (Essen, Germany). For the drug release studies 0.1 M hydrochloric acid (HCl), Hanks' balanced salt solution (99.015 mol% water, 0.95% Hanks' balanced salt and 0.035% sodium bicarbonate adjusted to pH 6.3 using 0.1M HCl), and phosphate buffered saline (PBS, pH 7.4) were used to simulate the pH conditions of the stomach [12, 14], small intestine [14], and colonic region, respectively. All components for the release media were purchased from Sigma Aldrich (Dorset, UK). Sodium taurocholate (ST) (10 mM) was used as a model bile salt in the small intestine buffer [15] and *β*-glucosidase (4% w/v, ≥ 24,000 units/100 mL) from almond emulsin (Sigma Aldrich) was added to the PBS as its chitinase activity is considered to be representative of that occurring in the colonic region [16–18]. All other chemicals and solvents used were purchased from Fisher Scientific and used as received.

### 2.2. Preparation Methods

#### 2.2.1. Formulation of Liposomes and Subsequent Coating with Chitosan

Liposomes were prepared using EPC and CH in the molar ratio 7 : 2, with DCP comprising 10% of the total lipid for anionic formulations. The conventional thin film hydration method [19] was used to produce multilamellar vesicles (MLVs), which were then extruded to produce large unilamellar vesicles (LUVs) for the study. Briefly, the lipids were dissolved in 5 mL chloroform in a 50 ml round bottom flask. The chloroform was then removed using a rotary evaporator, leaving a thin lipid film on the side of the flask which was then dried under nitrogen for 2 hours to remove trace chloroform. The film was then hydrated with an aqueous solution containing 1 mg/ml 5-ASA in PBS (pH7.4). During hydration the flask was agitated using a vortex mixer. Extrusion was carried out using an Avanti Lipid miniextruder through membranes with progressively smaller pores (1 *μ*m, 0.4 *μ*m and 0.2 *μ*m). Each sample was passed through each membrane fifteen times, producing vesicles with a narrow size distribution. Excess drug was removed through three cycles of centrifugation (63,000 relative centrifugal force (rcf)) and replacement of supernatant with PBS. The final pellet was then resuspended in 10 mL of PBS.

To prepare the coated liposomes equal volumes of liposomal suspension and aqueous solution of chitosan of various concentrations (0.25, 0.5, 1, 2 and 3% w/v in 1% acetic acid) were combined. Liposomal suspensions were added dropwise to the chitosan solution whilst under magnetic stirring, with the stirring being continued for a further 5 minutes [20–22]. The chitosan-coated liposomes were then left at 4°C for 24 hours to allow them to stabilise [23–25]. Excess chitosan was then removed by washing three times by centrifugation (63,000 rcf) and replacement of supernatant with 1% acetic acid.

#### 2.2.2. Encapsulation of Chitosan-Coated Liposomes within Eudragit S100 Microspheres

Chitosan-coated LUVs were encapsulated within Eudragit S100 microspheres using a double emulsion-solvent evaporation technique developed from previous work by Park et al. [26]. Eudragit S100 was dissolved in a solvent mixture of DCM:ethanol:propanol (5 : 6 : 4) to produce a 6% solution (w/w). 5 mL of the organic solution was added to a water phase comprising 0.8 mL of the chitosan-coated LUV suspension and 0.2mL polysorbate 20 (3%w/w) which had previously been vortex mixed (2,400 rpm, Fisherbrand FB15024). The primary emulsion [W_1_/O] was then formed by homogenising the solution for 2 minutes at 7,400 rpm (IKAT25 homogeniser, Fisher Scientific). The primary emulsion was then poured into 100 mL 1% PVA whilst under magnetic stirring at 125 rpm, thus creating the double emulsion [W_1_/O/W_2_]. The LIMs were magnetically stirred for 3 hours for subsequent polymer hardening and solvent evaporation. LIMs were then harvested by washing and vacuum filtration (filter membrane 1.6 *μ*m) with 200 mL distilled water to remove any excess surfactant.

### 2.3. Characterisation of Formulations

#### 2.3.1. Zeta Potential

Changes in dispersion zeta potential as a function of chitosan concentration were determined through electrophoretic mobility measurements (Zetamaster, Malvern Instruments, UK). Briefly, 500 *μ*L of the liposome/polymer suspensions (from Section 2.2.1) were diluted with 20 mL of distilled water (pH < 7) before introducing to the electrophoresis cell. Ten measurements were taken at 25°C on three samples from three independent formulations.

#### 2.3.2. Size Distribution

Vesicle size and size distribution before and after coating with chitosan were measured using wet laser diffraction particle sizing (Mastersizer 2000 connected to a Hydro SM small volume sample dispersion unit, Malvern Instruments, UK). Measurements were carried out in distilled water in which the polymer was not soluble. Three independent formulations of each preparation were each measured 5 times. 

#### 2.3.3. FITC Labelling of Chitosan and Subsequent Fluorescence Microscopy

To visualise the chitosan coating layer on the liposomes a method used by Amin et al. [24] was adopted. FITC-labelled chitosan was synthesized by adding 100 mL dehydrated methanol followed by 50 mL of FTIC in methanol (2.0 mg/mL) to 100 mL of chitosan (1% in 0.1 M CH_3_COOH) in the dark and at ambient temperature. After 3 hours of magnetic stirring at 500 rpm, the labelled polymer was precipitated in 0.2 M NaOH. The precipitate was pelleted at63,000 rcf (10 min) and washed with methanol-water (70:30, v/v) three times, at which point no fluorescence was observed in the supernatant. The labelled chitosan was then redissolved in 20 mL of 0.1 M acetic acid creating a solution of suitable concentration for subsequent liposome coating (Section 2.2.1). 

#### 2.3.4. Cryo-Scanning Electron Microscopy (Cryo-SEM)

LIMs were suspended in 5 M sucrose solution to maintain a stable suspension of microspheres and to avoid the sample settling. Drops of the LIM suspension were dispersed into the wells of the sample holder. The sample holder was then quenched in liquid nitrogen under vacuum conditions. Fracturing of the samples was conducted within the preparation chamber, through the use of a fine blade, using a Polaron Polar Preparation 2000 attached to a Phillips XL 30 Environmental Scanning Electron Microscope (ESEM). The samples were then coated with gold to increase conductivity and transferred into the ESEM chamber. Images were taken at a maximum voltage of 5.0 kV to reduce temperature fluctuations associated with higher voltages, with the instrument maintained at −180°C by the periodic addition of liquid nitrogen to the cooling chamber. 

#### 2.3.5. Degradation of LIMs in GI Tract Conditions

An SEM imaging study was conducted to assess the stability of the LIM formulation in the media representative of the GI tract conditions outlined in Section 2.1. LIMs were placed in each of the release media at concentrations equivalent to the drug release trials outlined in Section 2.4 and agitated in an incubator maintained at 37°C. At predetermined time points, samples were taken, centrifuged (63,000 rcf for 10minutes), the supernatant discarded and the pellet left to dry for 48 hours at room temperature. The dried pellet was then coated with platinum (Emscope SC500 sputter coater, 2 minutes) and subsequently imaged using scanning electron microscopy with a Jeol 6060 SEM under vacuum conditions.

### 2.4. Drug Release Studies

Drug release studies with chitosan-coated liposomes and LIMs were conducted in each of the different media described in Section 2.1. 50 mg of LIMs were inserted into a prehydrated 14,000 MW cutoff (MWCO) dialysis membrane (Biodesign, NY) with 5 mL of release media, and sealed. The membrane was then placed in a 250 mL conical flask containing 100 mL of the release media. The flasks were then placed in an incubator maintained at 37°C and agitated. Sink conditions were maintained throughout each experiment. Aliquots of 1 mL were removed at regular time intervals and replaced with 1mL of fresh, preheated buffer. The removed aliquot was then analysed for 5-ASA by UV spectrophotometry against a standard curve (*R* ^2^ > 0.99) obtained at *λ* = 330 nm. All measurements were taken against reference samples of an appropriate release medium. The containment of the formulations within a dialysis membrane allowed their removal from one medium and sequential exposure to another in a manner simulating progression through the GI tract. For each stage of the release study the sample was spun down (63,000 rcf for 10 minutes) and then resuspended with the next simulated GI tract fluid. During the trials in the colonic conditions it was observed that the *β*-glucosidase could also digest the cellulose dialysis membrane, thereby interfering with the absorbance readings necessary to quantify the drug release. However, an experiment was conducted which showed it took longer than 6 hours for this to take place and therefore the membrane was changed every 6 hours in the colonic buffer. 

For each formulation a sample was removed after preparation and the initial total drug loading quantified. This involved removing each layer of the LIMs to release the drug within the liposomes. The LIMs were initially exposed to the solvent mixture used in microsphere production (DCM:ethanol:propanol) to dissolve the Eudragit S100, then centrifuged at 26,000rpm (63,000 relative centrifugal force for 10 minutes) to pellet the chitosan-coated liposomes. The supernatant was analysed for drug using UV spectrophometry. The chitosan layer was then removed by exposing the liposomes to acetic acid. Once again, the sample was centrifuged and the supernatant analysed for drug. The final stage involved lysing of the liposomes and quantification of entrapped drug. This method for determining drug loading allowed the spatial location of the drug to be confirmed and thus provided evidence that intact, drug-loaded liposomes had been entrapped within the microspheres. Less than 2% of total drug was found in the microsphere layer and less than 5% was released following chitosan solubilisation.

## 3. Results and Discussion

### 3.1. Chitosan-Coated Liposomes

Table 1 shows vesicle zeta potential as a function of polymer (chitosan) concentration for both neutral and negatively charged liposomal formulations. An increase in zeta potential was observed with the inclusion of chitosan. For both anionic and neutral liposomal formulations no further change in zeta potential was observed once the concentration of the chitosan coating solution had reached 1% indicating that vesicle surfaces were saturated at this point. Further evidence that a coating layer had formed was also obtained through laser diffraction particle size measurements; d_50_ values for uncoated anionic and neutral liposomes were 0.148 (±0.003) *μ*m and 0.155 (±0.004) *μ*m, increasing to 0.187 (±0.007) *μ*m and 0.196 (±0.006) *μ*m for coated formulations. Both of these methods have previously been used to investigate the development of a chitosan coating layer on anionic and neutral liposomes [21–23, 27, 28]. It is thought that electrostatic interactions dominate in the coating of anionic liposomes with cationic chitosan [21, 22] while hydrophobic interactions are important for neutral liposomes, with hydrogen bonding occurring between the chitosan and phospholipid head groups of the lipid bilayer [22].

Figure 1 shows fluorescence microscope images comparing (a) neutral and (b) negatively charged liposomes when coated with a 1% solution of FITC-labelled chitosan. This use of fluorescence microscopy to characterise chitosan coating has not been extensively reported, and these images are some of the clearest found in the literature and further support the presence of the coating layer. 

The neutral liposomal formulation shows a number of discrete and coated liposomes (Figure 1(a)). Many more such vesicles were observed prior to capturing the image, but due to bleaching they are not present on the image. The layer itself is uniform in appearance, indicating that the vesicle surface is saturated with chitosan. This observation is consistent with the zeta potential measurements. The black centres of the vesicles indicate where the chitosan has not been able to penetrate, i.e., the aqueous core of the liposomes. For negatively charged liposomes, an agglomeration of coated vesicles is seen (Figure 1(b)). Such agglomeration is consistent with charge mosaic theory [23, 28, 29]. This theory states that the interactions between charged uncoated liposomes and partially coated liposomes (where the coat is of opposite charge) can lead to the agglomeration of particles and therefore the production of larger liposome/chitosan complexes. Given that the charged liposomal formulations tended to agglomerate in this way, it was decided to use neutral liposomes in the LIM formulations.

The use of cryo-SEM further indicated the presence of a chitosan coating layer around MLV formulations made under equivalent coating conditions described for LUVs (Figure 2). (MLVs were used here as their larger size and presence of multiple bilayers makes liposome identification easier). For the uncoated liposome (Figure 2(a)) bilayers are observed and the internal aqueous core can also be seen at the centre of the liposome. In comparison, the coated liposomes (Figure 2(b)) have a solid outer shell which is an indication of the chitosan coating. 

Overall, there was substantial evidence to indicate that the liposomal formulations were successfully coated with chitosan (Table 1 and Figures 1 and 2). As one of the reasons to coat the liposomes was to protect them during encapsulation, further studies to prove their stability in conditions representative of LIM production were completed. Chitosan-coated liposomes in aqueous suspension were exposed to the solvent mixture used during microsphere production (DCM:ethanol:propanol) and homogenised (Section 2.2.2). Subsequent centrifugation (63,000 rcf) and supernatant analysis revealed that no drug leakage had occurred, with light microscopy confirming the presence of intact liposome vesicles (not shown).

### 3.2. LIM Production and Characterisation

LIMs have been described previously, but not for colonic drug delivery. Feng et al. [30] produced microspheres using the biodegradable block copolymer poly (lactic acid), poly(ethylene glycol), and poly(lactic acid) (PLA-PEG-PLA) which provided a slow release of chitosan-coated liposomes of approximately 60% in 30 days with a view to solve the problems associated with DNA uptake at the liver for gene therapy. Park et al. [26] produced LIMs using alginate or extracellular polysaccharide to provide protection for liposomes through the stomach which then released cyclosporine A-loaded liposomes in the small intestine. 

LIM production in this study was based on the classic emulsification-solvent evaporation technique for microsphere production [31–34] involving the formation of a [W_1_/O/W_2_] emulsion. Given that the chitosan-coated liposomes were dispersed in the internal phase [W_1_] it was expected that they would be internalised within the microspheres that form as solvent diffuses out of the [O] phase into the continuous [W_2_] phase. The presence of polysorbate 20 was expected to facilitate containment of liposomes within the [W_1_] phase rather than allowing them to partition into the [O] phase. 

Figure 3 shows cryo-SEM images comparing the internal structure of an empty microsphere (produced with no liposomes present) with that of a LIM particle. The empty microsphere (Figure 3(a)) has a hollow interior with an outer shell. In Figure 3(b) the presence of the chitosan-coated LUVs can be clearly seen within the microsphere. The internal structure of the LIMs is similar to that observed by both Feng et al. [30] and Park et al. [26]. 

### 3.3. LIM Degradation and * In Vitro * Drug Release

Degradation studies were completed to observe the stability of the LIMs in each of the release media (Figures 4, 5, and 6).  Figure 4 shows SEM images of LIMs prior to and after two hours of exposure to 0.1 M HCl in conditions representative of the drug release trials. Two hours is generally accepted as the maximum transit time through the stomach [35] and therefore provides a good indication of gastric stability. No difference can be seen between the two images in Figure 4, with LIM surface morphology and structure remaining the same after the 2 hours. Similarly in conditions representative of the small intestine no visible change is observed in LIM appearance after three hours of exposure to the pH 6.3 buffer containing sodium taurocholate (Figure 5). 

In comparison, the images for LIMs subject to simulated colonic conditions show that degradation has commenced by 30 minutes (Figure 6(a)) with clear indication of changes on the surface of the microspheres. The onset of degradation for Eudragit S100 films has been shown to occur within minutes at pH > 7 [36, 37], indicating that microsphere degradation is likely begin as soon as the pH reaches 7 (e.g., around the ileocaecal junction). Lee et al. [37] observed 90% drug release from Eudragit S100 after 1 hour in pH 7.4 PBS indicating the rapid degradation of Eudragit S100, similar to that observed in the present study. It is therefore likely that the transit time in conditions above pH 7 would be sufficient to degrade the microspheres and allow liposome release within the colon. However, where there is doubt that the pH threshold will be reached *in vivo, *it has been shown that combining Eudragit S100 and L100 leads to a lower pH solubilisation point, allowing for release in patients with a reduced large intestine pH [38].

The degradation process continued with significant microsphere breakdown observed after 2 hours (Figure 6(b)). By 6 hours discrete microspheres were no longer visible (Figure 6(d)). Samples taken after 8 hours resulted in no polymer pellet being formed after centrifugation indicating that the Eudragit S100 was fully solubilised by this point. A small amount of lipid residue could be observed after centrifugation which was assumed to be the released liposomes. 

The drug release profiles comparing chitosan-coated LUVs and LIMs are shown in Figure 7. From the release profile for chitosan-coated LUVs it is evident there is a need for the gastro-resistant coating as chitosan is soluble in acidic conditions and therefore drug release can be observed within the first 30 minutes of exposure to the stomach conditions. Around 60% of the 5-ASA is released prior to reaching the large intestine and therefore the liposomes alone would not be a suitable delivery vehicle. In contrast, very little drug release was observed from LIMs in the stomach and small intestine conditions with subsequent drug release being observed in the colonic conditions. Labels on the LIM release curve in Figure 7 refer to the corresponding SEM images which indicate the stage of microsphere degradation at each point. As expected, for the stages where the microspheres are seen to be intact (2 hours in gastric conditions, 3 hours in small intestine conditions), very little drug release is observed therefore indicating that the LUVs are maintained within the microspheres. Importantly, the formulation was resistant to attack by bile salts, which was not previously observed when liposomes were coated directly with Eudragit S100 [10]. Once microsphere degradation occurs (within 30 minutes of exposure to large intestine conditions) significant drug release commences. From the SEM images it was shown that very few microsphere structures remained after 6 hours of exposure to the large intestine conditions, which corresponds to 11 hours on the drug release curve, indicating that most, if not all, of the liposomes would be exposed at this point and therefore chitosan solubilisation and subsequent drug release can occur. A number of studies [17, 18, 35] have proposed that the chitosan coating will be degraded *in vivo*, by observing *in vitro* studies using rat caecal contents and *β*-glucosidase to represent conditions created by the human microflora. 

## 4. Conclusion

A liposomal formulation suitable for lower GI tract targeting and oral administration could open up new opportunities in both local and systemic drug delivery. Here, a LIM system comprising features that would allow colonic targeting based on regional pH and enzymatic conditions was shown to remain intact throughout simulated stomach and small intestine conditions, preventing premature drug release. Upon exposure to simulated large intestine conditions, microsphere degradation was shown to occur within 30 minutes leading to substantial drug release well within the average transit time associated with the colon. The formulation has therefore demonstrated, *in vitro*, that it has properties necessary for direct targeting to the colon. 

## Figures and Tables

**Figure 1:** Fluorescence microscopy images of (a) neutral liposomes and (b) negatively charged liposomes coated with FITC labelled chitosan.

**Figure 2:** Cryo-SEM images of (a) uncoated MLVs and (b) MLVs coated with a 1% chitosan solution.

**Figure 3:** Cryo-SEM images of (a) an empty Eudragit S100 microsphere (water as the internal aqueous phase) and (b) a LIM particle.

**Figure 4:** SEM images showing LIMs suspended in pH 1.4 HCl for (a) 0 and (b) 2 hours.

**Figure 5:** SEM images showing LIMs suspended in pH 6.3 Hanks' buffer containing sodium taurocholate (10 mM) for (a) 0 and (b) 3 hours. Scale bar in (a) = 50 *μ*m and in (b) = 100 *μ*m.

**Figure 6:** SEM images showing LIMs suspended in pH 7.4 PBS containing *β*-glucosidase for (a) 0.5, (b) 2, (c) 4, and (d) 6 hours.

**Figure 7:** Drug release profiles comparing chitosan-coated liposomes (open symbols) with LIMs (black symbols) in simulated GI tract conditions. Each point represents the overall average from three independent experiments ± the standard error of the mean. The figure labels refer to the SEM images which show LIM structure at the various stages throughout the drug release trial.

**Table 1:** The effect of chitosan addition on the zeta potential of anionic and neutral LUVs. Each value represents the overall mean from three independent formulations ± the standard error of the mean.

	Chitosan concentration in coating solution (% w/v)					
	0.00	0.25	0.50	1.00	2.00	3.00
Anionic	−37.8 ± 0.8	−26.5 ± 3.9	16.1 ± 1.7	37.1 ± 1.4	37.1 ± 2.2	40.2 ± 2.4
Neutral	−0.1 ± 1.4	15.4 ± 2.1	23.6 ± 2.2	39.3 ± 2.6	39.4 ± 1.0	35.8 ± 2.6
